# mRNA Network: Solution for Tracking Chemotherapy Insensitivity in Small-Cell Lung Cancer

This article has been retracted.

**DOI:** 10.1155/2021/2105176

**Published:** 2021-09-28

**Authors:** Peixin Chen, Shengyu Wu, Jia Yu, Xuzhen Tang, Chunlei Dai, Hui Qi, Junjie Zhu, Wei Li, Bin Chen, Jun Zhu, Hao Wang, Sha Zhao, Hongcheng Liu, Peng Kuang, Yayi He

**Affiliations:** ^1^Department of Medical Oncology, Shanghai Pulmonary Hospital, Tongji University Medical School Cancer Institute, Tongji University School of Medicine, Shanghai 200433, China; ^2^Medical School, Tongji University, Shanghai 200433, China; ^3^Oncology and Immunology BU, Research Service Division, WuXi Apptec, Shanghai, China; ^4^Department of Surgery, Shanghai Pulmonary Hospital, Tongji University, Tongji University School of Medicine, Shanghai 200433, China; ^5^Department of Medical Oncology, The First Affiliated Hospital of Nanchang University, Nanchang 330006, China

## Abstract

**Background:**

Small-cell lung cancer (SCLC) has poor prognosis and is prone to drug resistance. It is necessary to search for possible influencing factors for SCLC chemotherapy insensitivity. Therefore, we proposed an mRNA network to track the chemotherapy insensitivity in SCLC.

**Methods:**

Six samples of patients with SCLC were recruited for RNA sequencing. TopHat2 and Cufflinks were used to make differential analysis. Functional analysis was applied as well. Finally, multidimensional validation was applied for verifying the results we obtained by experiment.

**Results:**

This study was a trial of drug resistance in 6 SCLC patients after first-line chemotherapy. The top 10 downregulated genes differentially expressed in the chemo-insensitive group were SERPING1, DRD5, PARVG, PRAME, NKX1-1, MCTP2, PID1, PLEKHA4, SPP1, and SLN. Cell-cell signaling by Wnt (*p*=6.98*E* − 21) was the most significantly enriched GO term in biological process, while systemic lupus erythematosus (*p*=6.97*E* − 10), alcoholism (*p*=1.01*E* − 09), and transcriptional misregulation in cancer (*p*=0.00227988) were the top three ones of KEGG pathways. In multiple public databases, we also highlighted and verified the vital role of glycolysis/gluconeogenesis pathway and corresponding genes in chemo-insensitivity in SCLC.

**Conclusion:**

Our study confirmed some SCLC chemotherapy insensitivity-related genes, biological processes, and pathways, thus constructing the chemotherapy-insensitive network for SCLC.

## 1. Introduction

Small-cell lung cancer (SCLC), as a kind of neuroendocrine tumor, remains one of the most deadly cancers [1]. Surgery for SCLC is limited to very early stages [2]. Chemotherapy is the first-line and second-line standard treatment for SCLC [3]. Etoposide/cisplatin (EP) [4] and etoposide/carboplatin (EC) [5] were clinically used for limited disease (LD) SCLC and extensive disease (ED) SCLC. Cisplatin/irinotecan was applied for LD-SCLC (JCOG0202) [6]. Topotecan [7], irinotecan [8], gemcitabine [9], and many others are often chosen for relapsed or refractory SCLC. For patients with SCLC, there are some clinical trials to investigate more effective combination therapy regimens. For example, the TORG 0604 trail illustrated the efficacy and safety of carboplatin combined with irinotecan and sequential thoracic radiotherapy (TRT) for patients with LD-SCLC [10]. For patients with ED-SCLC, the ECOG-ACRIN 2511 study aimed to evaluate the efficacy of EP combined with veliparib or placebo [11]. Nevertheless, there are still some SCLC patients insensitive to chemotherapy, which affect the clinical prognosis seriously [12, 13]. In the CONVERT trail, circulating tumor cells were used for efficacy evaluation and prognosis prediction [14]. However, the mechanisms of chemotherapy resistance in SCLC are complex [13, 15]. As a result, it is necessary to search for more possible influencing factors for SCLC chemotherapy insensitivity.

Messenger RNA (mRNA) is transcribed from DNA and carries the corresponding genetic information to provide the necessary information for the next translation into protein [16]. Previous studies have suggested strong association with mRNAs and drug resistance based on RNA sequencing (RNA-Seq). For instance, paclitaxel resistance is correlated with ABCB1 mRNA expression [17]. Other mRNAs such as FBXW7 were documented to be resistant to gefitinib and promoted tumor development [18]. Therefore, we proposed that mRNAs play a role in SCLC chemotherapy insensitivity.

This study set out to construct the mRNA network of chemotherapy insensitivity in SCLC. We considered the reasons of drug insensitivity from four aspects: the genes, the biological process, the KEGG pathways, and mutations of drug targets. Based on RNA-Seq and differential analysis, the upregulated and downregulated genes were identified. After that, Gene Ontology (GO) and Kyoto Encyclopedia of Genes and Genomes (KEGG) analyses were performed. We also did multidimensional validation to explore the hypothesis in view of the experiment.

To our knowledge, this study proposed a new direction of chemical resistance in SCLC. Some genes and pathways which have never revealed their function before were shown in our study. It thus provides new strategies for treatment henceforth. Importantly, multiple public databases were fully used to further verify the results we obtained by experiment.

## 2. Methods

### 2.1. Data Acquisition

After recruiting patients by lung biopsy for diagnosis from October 2018 to February 2019 in Shanghai Pulmonary Hospital, 6 male SCLC patients remained finally. All of them signed informed consent. The experimental protocol acquired Shanghai Pulmonary Hospital Ethics Committee permission [19].

### 2.2. RNA-Seq Analysis

Prior to sequencing library, total RNA needed to be extracted right after the section was diagnosed as SCLC by pathologists. It was extracted from fresh frozen SCLC tissues with an RNeasy 96 Universal Tissue Kit (Qiagen, Gaithersburg, MD, USA). After RNA isolation, the extraction effect was detected by agarose gel electrophoresis (Thermo Scientific, Bioanalyzer 2100; Agilent Technologies, USA). A Nano-Drop spectrophotometer (Nano-Drop 1000 Spectrometer) was next used to determine the quality and concentration of the total RNA (1.7 < OD260/OD280 < 2.0).

The next step in this process was construction of sequencing library. The double-stranded cDNA was synthesized by reverse transcription reaction, which added “A” in the 3′ end (Illumina, San Diego, CA, USA). Following this process, Illumina TruSeq RNA was constructed.

Following the use of electrophoresis to extract double-stranded cDNA fragment, suitable fragments were isolated. Then, DNA cluster amplification was carried out by quantitative polymerase chain reaction. The DNA amplicons were linearized into a single strand. Finally, high-throughput RNA-Seq was performed using the Illumina HiSeqTM 2000 platform [19].

### 2.3. Utility of Differential Analysis

TopHat2 [20] and Cufflinks [21] were used to analyze RNA-Seq data. RNA-Seq reads were mapped to the reference genome by TopHat2. Afterwards, multiple sequence alignment and transcriptional abundances were performed by Cufflinks. Therefore, differentially expressed genes (DEGs) could be identified.

Based on Cufflinks package (Cufflinks, Cuffmerge, Cuffcompare, and Cuffdiff), transcripts were assembled. Then, transcript assemblies were compared to annotation and merged. Finally, DEGs were found. We chose mean fold change (FC) as the gene expression relative abundance. On completion of analysis in Cufflinks package, the paired *t*-test was executed for significant difference analysis in different groups.

### 2.4. Functional and Pathway Enrichment Analyses

Functional enrichment analysis like GO [22–24] and pathway enrichment analysis such as KEGG enrichment analysis [25, 26] were employed. R version 2.15.1 (http://www.r-project.org.) was utilized for differential gene visualization. *p* ≥ 0.05 was not statistically significant.

### 2.5. Multidimensional Validation

In support of our experimental result, multidimensional validation was employed for minimizing bias. AmiGo2 software was selected for further GO analysis (http://amigo.geneontology.org/amigo/landing.). KEGG Pathway database [27] was in use for verifying significantly enriched pathways in this study. Pathway Card [28] was then applied for the main genes in the KEGG pathway. The effect of those main genes was discussed in some public databases from tissues (The Genotype-Tissue Expression (GTEx) [29], PROGgeneV2 [30], cBioportal [31], and The Human Protein Atlas [32]), cells (Cancer Cell Line Encyclopedia (CCLE) [33] and Oncomine [34]), and molecules (Metascape [35] and String [36]) (Figure 1).

All the processes are shown in Figure 2.

## 3. Results

### 3.1. Clinical Characteristics of SCLC Patients

This study was a trial of drug resistance in 6 SCLC patients after first-line chemotherapy. The average age was 64.2. All these patients were males and smokers. Two of them were LD-SCLC, and the rest were in the stage of ED. Among them, four patients had tumor metastasis while two did not. Only one of them received the treatment plan as EP. Others adopted EC. One half of them were identified as partial response (PR), and the other half were progressive disease (PD) or stable disease (SD) [19].

### 3.2. Features of RNA-Seq Results

We chose total throughput, counted reads, left processed, right processed, and total mapped features as key points of analysis in RNA-Seq. All these data were not apparently different between the PR group and the SD + PD group.  Table 1 provides an overview of RNA-Seq features in two groups.

### 3.3. Differentially Expressed mRNAs

Based on R software, we analyzed all data and selected the DEGs. We also identified the absolute value of FC > 2 and *p* value by the paired *t*-test less than 0.05 as the criterion for differentially expressed mRNAs. The top 10 downregulated genes differentially expressed in chemo-insensitive (SD or PD) tissues compared to those in chemo-sensitive (PR) tissues were SERPING1, DRD5, PARVG, PRAME, NKX1-1, MCTP2, PID1, PLEKHA4, SPP1, and SLN (Table 2), whereas AC008763.3, DBX2, ZIC1, CHRM3, ZNF541, AGBL1, TNNI2, MTUS2, CCDC36, and STAG3 were the top 10 upregulated DEGs (Table 3).

### 3.4. GO Categories and KEGG Pathways

Three GO categories were applied for the PR and SD + PD groups in this research: cellular component (CC), biological process (BP), and molecular function (MF). The bar chart presented the count and description of the three GO functions (Figure 3). What stands out in CC was the axon part (GO: 0033267, *p*=2.42*E* − 25). The column height implied the number of genes in each term. After GO enrichment analysis, the results of top 10 GO terms are set out in Table 4. Cell-cell signaling by Wnt (GO: 0198738) was the most significantly enriched GO-BP function due to the minimum *p* value (*p*=6.98*E* − 21). Other enriched GO-BP functions identified were Wnt signaling pathway (GO: 0016055, *p*=1.18*E* − 20), Ras protein signal transduction (GO: 0007265, *p*=1.83*E* − 20), and other terms.

DMGs were assigned to KEGG pathways as well. The count of genes in each description can be clearly seen in Figure 4. The top 3 enriched KEGG pathways were systemic lupus erythematosus (hsa05322, *p*=6.97*E* − 10), alcoholism (hsa05034, *p*=1.01*E* − 09), and transcriptional misregulation in cancer (hsa05202, *p* = 0.00227988) (Table 5).

### 3.5. Multidimensional Validation

We chose AmiGo2 software to find the association between meaningful GO terms mentioned above. Except for two GO terms (GO: 0000982 and GO: 0033267), extensive interaction was found among enrolled GO terms and other GO terms. In the whole database, the location of top 10 GO terms mentioned in Table 4 was illustrated (Figure S1).

Considering the vital role of metabolism in cancer development, progression, and metastasis, on the basis of KEGG results, we put forward a hypothesis that the glycolysis/gluconeogenesis pathway might play a nonnegligible role in SCLC. To verify our hypothesis, firstly, KEGG Pathway database [37] was applied for the glycolysis/gluconeogenesis pathway (Figure S2). Then, glycolysis/gluconeogenesis pathway-related genes were demonstrated from Pathway Card [38]. Phosphoglycerate mutase 2 (PGAM2), phosphoglycerate kinase 1 (PGK1), glyceraldehyde-3-phosphate dehydrogenase (GAPDH), triosephosphate isomerase 1 (TPI1), and pyruvate kinase M1/2 (PKM) were the representative genes of the glycolysis/gluconeogenesis pathway. Subsequently, some databases were used for verifying the role of the pathway from three levels: tissue, cell, and molecule, for instance, GTEx (tissue) (Figure S3), PROGgeneV2 (tissue) (Figure S4), cBioportal (tissue) (Figures S5–S11), The Human Protein Atlas (tissue), CCLE (cell) (Figure S12), Oncomine (cell) (Figure S13), Metascape (molecule) (Figure S14), and String (molecule) (Figure S15). All of the details can be found in Tables S1 and S2. The expressions of PGAM2, PGK1, GAPDH, TPI1, and PKM were found in tumor tissues or cell lines (Figures S3–S15). In Figure S4, high GAPDH expression was linked to shorter overall survival (OS) in lung cancer (*p*=0.009812). In the cBioportal dataset, the survival analysis suggested that PKM mutation indicated poor prognosis (*p*=0.012, Figure S5). However, the sample size of the PKM mutation group was too small to fully reflect the relationship between mutation status of PKM and prognosis. Importantly, PGK1, GAPDH, and TPI1 were not mutated in tumor tissues as seen from the cBioportal dataset (Figure S5). In addition, in the cBioportal cohort with 81 clinical SCLC patients who owned RNA-Seq data, we explored the relationship between expression levels of main genes in the glycolysis/gluconeogenesis pathway and OS. As shown in Figure S6, high PKM expression was correlated with better prognosis (*p* < 0.0001). Then, the correlation between gene expression level and clinicopathologic features, including age, gender, smoking history, metastasis, and TNM staging, were estimated (Figures S7–S11). Overexpression of GAPDH, PGAM2, PGK1, and PKM was found in patients over the age of 65. In comparison with female patients, male patients with SCLC showed higher expression of PGAM2 and PGK1. GAPDH, PGAM2, PGK1, and PKM were also highly expressed in SCLC tissues from smokers. However, no significant results were found between gene expression and clinicopathologic features (both *p* > 0.05). The extensive connection among vital genes of the glycolysis/gluconeogenesis pathway was found (Figures S14 and S15). Overall, these multidimensional validations supported the view that the abnormal glycolysis/gluconeogenesis pathway had something to do with the chemotherapy insensitivity in SCLC.

In short, the network of DEGs in PR and SD + PD groups was constructed. Upregulated and downregulated DEGs in the PR group were found. DEGs-related GO terms and KEGG signaling pathways were also illustrated. Finally, scientific hypothesis was produced as follows: the chemotherapy insensitivity in SCLC was related to KEGG signaling pathways and GO terms, such as systemic lupus erythematosus, glycolysis/gluconeogenesis pathway, and cell-cell signaling by Wnt.

## 4. Discussion

Despite various treatments, systemic chemotherapy is still the main treatment for SCLC [39]. There are several clinical trials as well. For example, ipilimumab or placebo plus etoposide and platinum were used for efficacy and safety in ED-SCLC patients [40]. TORG 0604 was aimed at evaluating the effect of carboplatin combined with irinotecan and TRT in LD-SCLC [10]. In our study, EP and EC were supplied to these patients, respectively. The function of them was published in the JCOG 9702 trial. It revealed the curative effect in the elderly. EP was the traditional treatment and EC could be another alternative due to the similar palliative scores [41]. In recent years, much attention is paid to metronomic chemotherapy. Weekly paclitaxel is workable as a second-line treatment for recurrent SCLC [42]. However, the drug resistance of SCLC is inevitable although it is initially sensitive to chemotherapy [12, 13, 43]. With high recurrence rate, the exploration of factors for SCLC chemotherapy insensitivity is essential.

We proposed genes play a role in chemotherapy insensitivity. Previous studies have mentioned genes like MRP, MDR1 [44], EZH2 [45], and many others. In this paper, we identified the DEGs between PR and SD + PD group through RNA-Seq. It can sort, classify, and compare gene expression [46]. By detecting the transcription of mRNA, our study proved the downregulation of SPP1 was associated with chemotherapy resistance in SCLC, which was consistent with previous studies [47]. Recently, through in vivo and in vitro experiments, Tang et al. found that SPP1 induced non-small-cell lung cancer (NSCLC) progression and cisplatin resistance [48]. By RNA-Seq and differential analysis, we also found the correlation between downregulated genes like DRD5, PRAME, and SERPING1 and chemotherapy insensitivity. DRD5, which is associated with receptor-related signal transduction on cell surface [49], can inhibit tumor growth by promoting autophagic cell death [50]. There has been a considerable amount of investigation into PRAME. The expression of PRAME was correlated with tumor histology and smoking status [51]. It played an important role in the invasion [52] and metastasis [53] of lung cancer. For cancer patients, overexpression of PRAME was frequently correlated with poor prognosis [54, 55]. Furthermore, the low expression of SERPING1 represented poor prognosis in prostate cancer [56]. All these results suggested they were often downregulated in tumors and the downregulation led to tumor development and metastasis. However, there is limited report on their roles in drug resistance at present. This is what we need to further study in the future. STAG3 and CHRM3 upregulated in our research can be viewed as chemotherapy resistance-associated tumor genes. Mutations in STAG3 are usually associated with premature ovarian failure [57]. Downregulating the expression of STAG3 decreased the sensitivity of BRAF-mutant melanoma cells to inhibitors of BRAF [58]. CHRM3 seemed to be upregulated in gastric cancer patients who were responsive to ramucirumab [59]. Although they play the role of drug resistance in some cancers, there is still no clear evidence to demonstrate their relevant function in SCLC currently. Therefore, more researches are essential to clarify whether STAG3 and CHRM3 cause chemotherapy insensitivity in SCLC.

Functional and pathway enrichment analyses were also employed in our research. Based on GO and KEGG analysis for PR and SD + PD groups, biological characteristics of genes and the relationship between gene regulatory networks and gene function were discovered [60]. After GO analysis, we knew different activities in cells. In this case, SCLC chemotherapy insensitivity was mainly connected with cell-cell signaling by Wnt, Wnt signaling pathway, and Ras protein signal transduction on the cellular level. Afterwards, AmiGo2 software was applied for the associated genes in GO terms mentioned above and the location of GO terms in the whole database. Systemic lupus erythematosus, a KEGG pathway, was proved to be downregulated in the PR group. In recent years, mRNAs have been considered to be closely related to autoimmunity diseases [61]. Evidence showed the hierarchical association of systemic lupus erythematosus and various types of cancer, including lung cancer [62–65]. It was driven by gene region 6p21-22 and is strongly associated with lung cancer. However, this was correlated with squamous cell lung carcinoma [66]. Alcoholism was another significantly downregulated pathway in the PR group. Systemic lupus erythematosus and alcoholism also played a role in mitoxantrone insensitivity in NSCLC [67]. The related studies in SCLC are not sufficient at present. Our team has confirmed the two pathways above after analysis of long noncoding RNAs and microRNAs previously [19]. The same result in mRNA was proved this time.

Moreover, we found the aberrant glycolysis/gluconeogenesis KEGG pathway in SCLC chemotherapy resistance. With a *p* value less than 0.05, it was one of the significant pathways in our study. It belongs to pathway network for glucose metabolism, SuperPath [68, 69]. Just like any other type of cancer, SCLC cells use aerobic glycolysis as the main source of adenosine triphosphate [70]. Notably, higher total lesion glycolysis (TLG) is correlated with poorer prognosis of SCLC [71]. A-disintegrin-and-metalloproteinase 12-s (Adam12S), a protein related to tissue growth and development, promoted SCLC cell proliferation, migration, and invasion by upregulating the rate-limiting enzyme hexokinase 1 in glycolysis [72]. Reducing glycolysis can promote tumor invasion by SCLC cell population [73]. Monocarboxylate transporter 1 (MCT1) inhibitor called AZD3965 killed those glycolysis-dependent tumor cells through lactate transport regulation, especially in SCLC patients with tumor expression of MCT1 and lack of MCT4 [74]. Currently, the dependence of cancer cells on energy production by glycolysis has been well studied. There are also some research on the function of glycolysis and gluconeogenesis in chemotherapy insensitivity. Drug-resistant cancer cells showed higher glycolysis. Emerging evidence points to the abnormal glucose metabolism causing resistance to cancer therapy [75, 76]. And, targeting glycolysis pathway was considered as a new strategy to overcome drug resistance [77, 78]. The altered glycolysis may be connected with stem cell-like cancer [72]. Cancer stem cells were a kind of monoenergetic cell group existing in the tumor cell group and highly resistant to chemotherapeutic drugs [75]. In pancreatic cancer, L-type amino acid transporter 2 (LAT2) promoted glycolysis and reduced gemcitabine sensitivity by regulating glutamine-dependent mTOR [79]. Overexpression of FGFR4 can increase glucose metabolism and result in breast cancer chemical resistance [80]. In lung cancer, another important discovery was found. Hepatocyte growth factor (HGF) regulation by secreted lactate was the adaptive resistance that led to continuous resistance to tyrosine kinase inhibitors [81]. Although there has been substantial research on the mechanisms of cancer chemotherapy insensitivity, few are about gluconeogenesis. The mechanisms in SCLC also remain to be confirmed. To further verify the result of the abnormal glycolysis/gluconeogenesis pathway in SCLC chemical resistance by KEGG analysis, multidimensional validation was performed. We chose Pathway Card for the top five genes in the glycolysis/gluconeogenesis pathway. Then, we put them into some public databases to verify the pathway function. The result was the same as that in KEGG analysis.

Although these studies revealed important findings, they also had limitations. The findings were required to be carried out as in vivo and in vitro experiments. This is what we will do next. Furthermore, we must mention that the small sample size might have a certain impact on the result. A large number of patients with SCLC need to be investigated in the future.

## 5. Conclusion

Our study confirmed that genes such as SERPING1, DRD5, and PARVG were involved in SCLC chemotherapy response by complex biological processes. Pathways such as systemic lupus erythematosus, alcoholism, and glycolysis/gluconeogenesis were also involved.

## Figures and Tables

**Figure 1:** Some public databases from tissues, cells, and molecules.

**Figure 2:** Process of the total experiment.

**Figure 3:** Gene Ontology analysis from cellular component, biological process, and molecular function.

**Figure 4:** Kyoto Encyclopedia of Genes and Genomes enrichment.

**Table 1:** RNA-sequencing analysis results of 6 patients.

Features	PR group	SD + PD group	*p*
Total throughput, Mbp (mean ± SD)	5136 ± 1638	5295 ± 1056	NS
Counted reads, *M* (mean ± SD)	27.63 ± 7.20	26.61 ± 7.37	NS
Left processed, *M* (mean ± SD)	29.52 ± 9.25	29.87 ± 7.63	NS
Right processed, *M* (mean ± SD)	21.65 ± 8.31	22.94 ± 5.72	NS
Total mapped, *M* (mean ± SD)	35.16 ± 9.68	39.26 ± 12.82	NS

bp, base pair; *M*, millions; NS, nonsignificant; SD, standard deviation; PR group, partial response group; SD + PD group, stable disease and progressive disease group.

**Table 2:** The top 10 down-regulated DEGs in chemo-insensitive tissues compared to chemo-sensitive tissues.

Gene	Mean fold change	*p* value
SERPING1	0.000938518	7.38831*E* − 06
DRD5	0.001276883	1.40696*E* − 05
PARVG	0.001539754	0.000143271
PRAME	0.001617729	7.69512*E* − 05
NKX1-1	0.001806826	0.000243319
MCTP2	0.0018187	2.16951*E* − 06
PID1	0.001958718	0.00015673
PLEKHA4	0.002022778	3.68368*E* − 05
SPP1	0.002057895	0.00605997
SLN	0.002236008	0.000703164

DEGs, differentially expressed genes; SD, standard deviation.

**Table 3:** The top 10 up-regulated DEGs in chemo-insensitive tissues compared to chemo-sensitive tissues.

Gene	Mean fold change	*p* value
AC008763.3	474.0353333	0.001285241
DBX2	329.515	0.002263272
ZIC1	326.1616624	0.007815534
CHRM3	271.3690333	0.001168554
ZNF541	246.346	0.000100752
AGBL1	211.4909333	0.000734099
TNNI2	188.4115	0.002991354
MTUS2	160.068889	0.001778011
CCDC36	157.1693333	0.010546793
STAG3	149.0489868	3.94026*E* − 05

DEGs, differentially expressed genes; SD, standard deviation.

**Table 4:** Results of the enriched Gene Ontology (GO) term analysis.

GO ID	GO terms	GO categories	*p* value
GO: 0033267	Axon part	Cellular component	2.42*E* − 25
GO: 0198738	Cell-cell signaling by Wnt	Biological process	6.98*E* − 21
GO: 0016055	Wnt signaling pathway	Biological process	1.18*E* − 20
GO: 0007265	Ras protein signal transduction	Biological process	1.83*E* − 20
GO: 0150034	Distal axon	Cellular component	1.04*E* − 19
GO: 0007409	Axonogenesis	Biological process	1.40*E* − 19
GO: 0000982	Transcription factor activity, RNA polymerase II proximal promoter sequence-specific DNA binding	Molecular function	1.55*E* − 19
GO: 0098978	Glutamatergic synapse	Cellular component	9.12*E* − 19
GO: 0050804	Modulation of chemical synaptic transmission	Biological process	1.41*E* − 18
GO: 0099177	Regulation of trans-synaptic signaling	Biological process	2.90*E* − 18

**Table 5:** Results of the KEGG enriched pathway analysis.

KEGG ID	KEGG pathway	*p* value
hsa05322	Systemic lupus erythematosus	6.97*E* − 10
hsa05034	Alcoholism	1.01*E* − 09
hsa05202	Transcriptional misregulation in cancer	0.00227988
hsa04950	Maturity-onset diabetes in the young	0.007478296
hsa04217	Necroptosis	0.008674735
hsa00260	Glycine, serine, and threonine metabolism	0.017168326
hsa00010	Glycolysis/gluconeogenesis	0.045907156
hsa05230	Central carbon metabolism in cancer	0.047129544
hsa01230	Biosynthesis of amino acids	0.054710337
hsa04540	Gap junction	0.072470106

KEGG, Kyoto Encyclopedia of Genes and Genomes.

## Data Availability

The shared sequencing data can be obtained from the corresponding author upon request via email (yayi.he@tongji.edu.cn) for clinical and practical reasons.

## Abbreviations

SCLC: Small-cell lung cancer
mRNA: Messenger RNA
GO: Gene Ontology
KEGG: Kyoto Encyclopedia of Genes and Genomes
GTEx: The Genotype-Tissue Expression
CCLE: Cancer Cell Line Encyclopedia
LD: Limited disease
ED: Extensive disease
EP: Etoposide plus cisplatin
EC: Etoposide plus carboplatin
PR: Partial response
PD: Progressive disease
SD: Stable disease
FC: Fold change
CC: Cellular component
BP: Biological process
MF: Molecular function
PGAM2: Phosphoglycerate mutase 2
PGK1: Phosphoglycerate kinase 1
GAPDH: Glyceraldehyde-3-phosphate dehydrogenase
TPI1: Triosephosphate isomerase 1
PKM: Pyruvate kinase M1/2
TLG: Total lesion glycolysis
Adam12S: A-disintegrin-and-metalloproteinase 12-s
LAT2: L-type amino acid transporter 2
OS: Overall survival.

## Supplementary Materials

Supplementary Materials Table S1: multidimensional external validation results based on multiple databases. Table S2: summary of multidimensional external validation results based on multiple databases. Figure S1: the association and location of top 10 GO terms in AmiGo2 software. Figure S2: the glycolysis/gluconeogenesis pathway in the chemo-insensitive group. Figure S3: main genes in the KEGG pathway by GTEx and the comparison in expression between all these genes. Figure S4: main genes in the KEGG pathway by PROGgeneV2: (A) PGAM2, (B) PGK1, and (C) GAPDH. Figure S5: mutation status of main genes in the KEGG pathway by cBioportal; correlation between mutation status of (A) PGAM2, (B) PGK1, (C) GAPDH, (D) TPI1, and (E) PKM and survival and gene expression. Figure S6: relationship between expression levels of main genes in the KEGG pathway and survival in cBioportal: (A) GAPDH, (B) PGAM2, (C) PGK1, and (D) PKM. Figure S7: relationship between expression levels of main genes in the KEGG pathway and age in cBioportal: (A) GAPDH, (B) PGAM2, (C) PGK1, and (D) PKM. Figure S8: relationship between expression levels of main genes in the KEGG pathway and gender in cBioportal: (A) GAPDH, (B) PGAM2, (C) PGK1, and (D) PKM. Figure S9: relationship between expression levels of main genes in the KEGG pathway and TNM staging in cBioportal: (A) GAPDH, (B) PGAM2, (C) PGK1, and (D) PKM. Figure S10: relationship between expression levels of main genes in the KEGG pathway and smoking history in cBioportal: (A) GAPDH, (B) PGAM2, (C) PGK1, and (D) PKM. Figure S11: relationship between expression levels of main genes in the KEGG pathway and metastasis (M) in cBioportal: (A) GAPDH, (B) PGAM2, (C) PGK1, and (D) PKM. Figure S12: main genes in the KEGG pathway by CCLE; the expression level of (A) PGAM2, (B) PGK1, (C) GAPDH, (D) TPI1, and (E) PKM in the CCLE database. Figure S13: main genes in the KEGG pathway by Oncomine; the different expressions of (A) PGAM2, (B) PGK1, (C) GAPDH, (D) TPI1, and (E) PKM in lung cancer in Oncomine database. Figure S14: network of enriched terms and protein-protein interaction network by Metascape: (A) colored by cluster ID, nodes that share the same cluster ID are typically close to each other; (B) colored by *p* value, terms containing more genes tend to have a more significant *p* value; (C) protein-protein interaction network and MCODE components identified in the gene lists. Figure S15: gene coexpression and protein-protein interaction network by String: (A) the gene coexpression map; (B) protein-protein interaction network about PGAM2, PGK1, GAPDH, TPI1, and PKM.
